# Genetic Polymorphism of Matrix Metalloproteinase-9 and Susceptibility to Myocardial Infarction: A Meta-Analysis

**DOI:** 10.1155/2022/5507153

**Published:** 2022-01-15

**Authors:** Beili Feng, Hengdong Li

**Affiliations:** ^1^Department of Cardiology, HwaMei Hospital, University of Chinese Academy of Sciences, Ningbo, Zhejiang, China; ^2^Ningbo Institute of Life and Health Industry, University of Chinese Academy of Sciences, Ningbo, Zhejiang, China

## Abstract

**Objective:**

Current findings on the association between MMP-9 rs3918242 and susceptibility to myocardial infarction (MI) are inconsistent, and their definite relationship is discussed in this meta-analysis.

**Methods:**

Eligible literatures reporting MMP-9 rs3918242 and susceptibility to MI were searched in PubMed, Cochrane Library, CNRI, and VIP using keywords such as “MMP-9”, “matrix metallopeptidase-9” and “myocardial infarction”, “acute myocardial infarction”, “AMI”, and “polymorphism”. Data from eligible literatures were extracted for calculating OR and corresponding 95% CI using RevMan 5.3 and STATA12.0.

**Results:**

Ten independent literatures reporting MMP-9 rs3918242 and susceptibility to MI were enrolled. Compared with subjects carrying CT&TT genotype of MMP-9 rs3918242, susceptibility to MI was lower in those carrying CC genotype (OR = 1.49, 95%CI = 1.19–1.86, *P* = 0.0004). Such a significance was observed in the overdominant (OR = 1.27, 95%CI = 1.14–1.41, *P* < 0.0001) and allele genetic models (OR = 1.43, 95%CI = 1.17–1.74, *P* = 0.0005) as well. This finding was also valid in the Asian population.

**Conclusions:**

Mutation on MMP-9 rs3918242 has a potential relevance with susceptibility to MI.

## 1. Introduction

Acute myocardial infarction (AMI) manifests as myocardial necrosis which resulted from acute, persistent ischemia and hypoxia in the coronary arteries. In the United States, there are 5 million people that visit the emergency department because of acute chest pain. More than 800,000 AMI cases each year are newly onset, and 27% of them die before arriving at the hospital [1]. In recent years, the incidence of AMI has an obvious rise. There are at least 500,000 newly onsets and 2 million present illness cases of AMI. Risk factors for MI include three major categories: unchangeable factors (age, gender, and family history), variable factors (smoking, alcohol, lack of exercise, poor diet, high blood pressure, diabetes, dyslipidemia, and metabolism syndrome), and emerging factors (abnormal levels of CRP, fibrinogen, CAC, homocysteine, lipoprotein (a), and LDL) [2, 3]. Current researches have defined that interactions between various environmental factors and certain genetic polymorphisms may lead to AMI [4, 5]. In recent studies, SNP genetic variants were closely related to AMI. Williams et al. found that a SNP in CRP (rs2592902) was closely linked to ischemic and recurrent stroke [6]. Further, myocardial infarction-associated SNP at 6p24 interferes with MEF2 binding and associates with PHACTR1 expression levels in human coronary arteries [7]. In short, it is necessary to find new SNP site which was closely related to AMI.

The matrix metalloproteinase (MMP) family is composed of 20 secretory or ectocellular enzymes that degrade extracellular matrix proteins, coagulation factors, lipoproteins, latent growth factors, chemokines, and cell adhesion molecules [8, 9]. MMP levels are mainly mediated by transcriptional regulation. Meanwhile, MMP activities are linked with the activation of MMP zymogen and TIMPs (tissue inhibitors of MMPs) [8, 9]. MMP levels in blood vessels and heart tissues are closely related to many cardiovascular diseases, including atherosclerosis, aneurysms, restenosis after angioplasty, and heart failure [10, 11]. MMP-9 is an important enzyme that degrades the main component of vascular basement membrane (type IV collagen) and is closely related to the occurrence and development of atherosclerosis [10, 12]. The promoter region of MMP-9 C-1562T (rs3918242) is believed to be linked with MI. So far, a considerable number of studies have been conducted to analyze the MMP-9 rs3918242 and MI, whereas their conclusions are controversial. This study is aimed at uncovering a precise involvement of MMP-9 rs3918242 in MI.

## 2. Materials and Methods

### 2.1. Literature Screening

Eligible literatures reporting MMP-9 rs3918242 and susceptibility to MI published before May 2019 were searched in PubMed, Cochrane Library, CNRI, and VIP. Keywords searched were as follows: “MMP-9”, “matrix metallopeptidase-9” and “myocardial infarction”, “acute myocardial infarction”, “AMI”, and “polymorphism”. Citations in the selected literatures were manually examined.

Full text of each literature was reviewed and its eligibility determined using the following inclusive criteria: (1) independent case-control studies analyzing hospital-based or population-based subjects without any language limitations, (2) adequate data provided to obtain genotype frequencies, (3) literatures reporting MMP-9 rs3918242 and susceptibility to MI; (4) genotype distribution in the controls in accordance to HWE (Hardy-Weinberg equilibrium), and (5) no repeated published data.

Exclusive criteria included the following: (1) reviews, comments, animal experiments, mechanism researches, and case reports; (2) repeatedly published articles; and (3) studies with inadequate data. The flow diagram of the publication selection is depicted in Figure 1.

### 2.2. Data Extraction

Data were independently extracted and analyzed by two researchers. Any disagreement was solved by the third researcher. Extracted data included first author, year of publication, country of publication, genotype number and distribution, and case number.

### 2.3. Statistical Processing

Heterogeneity test was conducted by calculating OR and the corresponding 95% CI with the *I*^2^ test and the *Q* test. The pooled OR in studies lacking the heterogeneity was calculated by the fixed-effects model; otherwise, a random-effects model was used. Sensitivity analysis was conducted by removing one study each time and analyzing the remaining in a combination way. The HWE of control genotype distribution was evaluated using the *χ*^2^ test, and *P* < 0.05 considered as inequivalent. Publication bias was evaluated by depicting funnel plots and quantified by Egger's test. Data analyses were conducted using RevMan 5.3 and STATA12.0 (London, UK).

## 3. Results

### 3.1. Baseline Characteristics of Eligible Literatures

At first, 556 relevant literatures were searched from online databases. 276 repeated literatures and 241 irrelevant ones were excluded after reviewing the titles and abstracts. The remaining 39 literatures were assessed in details. 12 literatures with irrelevant findings, 5 abstracts/meta-analyses, 4 nonpolymorphism researches, and 8 literatures lacking adequate data or full text were excluded. At last, 10 eligible literatures published from 2005 to 2017 were enrolled [11–20]. Baseline characteristics of them and HWE results of the controls were detailed (Table 1). A total of 3087 MI patients and 5019 healthy controls were involved. Serum samples were detected by PCR/PCR-RFLP/TaqMan.

### 3.2. Meta-Analysis Results

MMP-9 rs3918242 polymorphism and susceptibility to MI were analyzed using different genetic models. Heterogeneity existed in the dominant (*I*^2^ = 53%, *P* = 0.02) and allele genetic models (*I*^2^ = 52%, *P* = 0.03), rather than recessive (*I*^2^ = 13%, *P* = 0.33) and overdominant genetic models (*I*^2^ = 46%, *P* = 0.06). Pooled OR was calculated according to the heterogeneity results. Compared with subjects carrying CT&TT genotype of MMP-9 rs3918242, susceptibility to MI was lower in those carrying CC genotype (OR = 1.49, 95%CI = 1.19–1.86, *P* = 0.0004). In addition, subjects carrying TT genotype had higher susceptibility to MI than those carrying CT&CC genotype (OR = 1.54, 95%CI = 1.08–2.20, *P* = 0.02). Such a significance was observed in the overdominant (OR = 1.27, 95%CI = 1.14–1.41, *P* < 0.0001) and allele genetic models (OR = 1.43, 95%CI = 1.17–1.74, *P* = 0.0005) as well (Figure 2).

Subgroup analyses were conducted based on ethnicity. A significant association between MMP-9 rs3918242 polymorphism and susceptibility to MI in Asian population was identified in dominant (OR = 1.61, 95%CI = 1.26–2.06, *P* = 0.0001), recessive (OR = 3.34, 95%CI = 1.29–8.67, *P* = 0.01), overdominant (OR = 1.50, 95%CI = 1.16–1.92, *P* = 0.002), and allele genetic models (OR = 1.58, 95%CI = 1.26–1.99, *P* < 0.0001). Such an association in Caucasian population was only uncovered in dominant (OR = 1.20, 95%CI = 1.06–1.36, *P* = 0.003), overdominant (OR = 1.17, 95%CI = 1.03–1.33, *P* = 0.01), and allele genetic models (OR = 1.55, 95%CI = 1.07–2.24, *P* = 0.02), rather than recessive model (OR = 1.39, 95%CI = 0.03–3.28, *P* = 0.10) (Figures 3–6).

### 3.3. Sensitivity Analysis

No significant changes in pooled *P* and OR were observed after removing one single article for each time, demonstrating the robust results of our analysis.

### 3.4. Publication Bias

Funnel plots depicted a symmetrical shape in the four genetic models (Figure 7). Egger's test clarified no significant difference in publication bias in allele (*t* = 1.44, *P* = 0.188), overdominant (*t* = 1.70, *P* = 0.128), recessive (*t* = 0.68, *P* = 0.528), and dominant genetic models (*t* = 1.67, *P* = 0.134), as well as subgroup analyses (data not shown).

## 4. Discussion

MMPs are a family of Zn^2+^-dependent neutral proteases that degrade and reshape extracellular matrices, maintain the homeostasis of extracellular matrices, and participate in pathological and physiological processes in humans. MMP-9 is the active enzyme in MMP family with the largest molecule size of all members. It mediates the formation, development, and rupture of atherosclerotic plaques by mediating metastasis, viability, apoptosis, and extracellular matrix remodeling of vascular smooth muscle cells [21, 22]. Studies have found that elevated levels of MMPs are closely associated with the development of unstable angina and AMI [23, 24]. Zouridakis et al. [25] analyzed the data from 124 patients with stable angina and demonstrated that MMP-9 is an independent predictor of atherosclerosis progression. Another study found that MMP-9 is one of the key factors affecting plaque stability and rupture [26].

MMP-9 contains 13 exons and 12 introns. The substitution of C in the promoter region -1562 of MMP-9 by T can change its activity. Morgan et al. [27] reported that the affinity of the MMP-9 gene nucleoprotein of the -1562T allele carrier is markedly higher than that of the C allele carrier. Promoter activity is higher in the population carrying MMP-9 -1562T relative to those carrying MMP-9 -1562C, indicating the influence of MMP-9-1562C>T polymorphism on the onset of MI.

Our findings illustrated higher frequency of MMP-9 T-base mutation in MI patients than that in healthy controls no matter in the whole population or different ethnicities. Higher susceptibility to MI was uncovered in people carrying T allele of MMP-9 (TC+CC) compared with those carrying CC genotype in both Asian and Caucasian population. Consistently, Wang et al. [28] analyzed 7 articles published from 1999 to 2010, involving 4473 MI patients and 3343 healthy controls. They pointed out the involvement of MMP-9 polymorphism in MI risk. Another meta-analysis demonstrated that MMP-9 C-1562T is only associated with MI onset in East Asian population rather than Western population [29]. Here, three enrolled articles were conducted in Caucasian population. Such an association in Caucasian population was only uncovered in dominant (TT & CT *vs.* CC), overdominant (CT *vs.* CC & TT), and allele genetic models (C allele *vs.* T allele).

Some limitations were present in this paper. Firstly, MMP-9 polymorphism may be interacted with unknown or well-known risk factors of MI, such as hypertension, diabetes, dyslipidemia, and previous coronary artery disease. Secondly, genotype distribution of MMP-9 failed to be calculated owing to a small sample size. Thirdly, literatures published in other languages were excluded. Fourthly, gender and other factors in MI patients should be taken into consideration. In summary, there was a lot of work that need to be done to confirm that the SNP in MMP-9 was a very key factor for AMI.

## 5. Conclusions

Collectively, MMP-9 rs3918242 had a potential relevance with susceptibility to MI. Our findings required to be validated in a multicenter hospital with larger sample size.

## Figures and Tables

**Figure 1:** Flow diagram of the publication selection process.

**Figure 2:** Forest plots demonstrating the association between MMP-9 polymorphism and susceptibility to myocardial infarction.

**Figure 3:** Forest plot of the meta-analysis of the association between MMP-9 C-1562T (rs3918242) and susceptibility to myocardial infarction in different ethnic subgroups using a dominant genetic model.

**Figure 4:** Forest plot of the meta-analysis of the association between MMP-9 C-1562T (rs3918242) and susceptibility to myocardial infarction in different ethnic subgroups using a recessive genetic model.

**Figure 5:** Forest plot of the meta-analysis of the association between MMP-9 C-1562T (rs3918242) and susceptibility to myocardial infarction in different ethnic subgroups using an overdominant genetic model.

**Figure 6:** Forest plot of the meta-analysis of the association between MMP-9 C-1562T (rs3918242) and susceptibility to myocardial infarction in different ethnic subgroups using an allele genetic model.

**Figure 7:** Publication bias on polymorphisms of MMP-9 rs3918242 and susceptibility to myocardial infarction.

**Table 1:** Baseline characteristics of eligible literatures.

Author	Year	Country	Journal name/ publication origin	Genotyping methods	SNP loci (*P*_HWE_)	Sample size	Control	Sample
Chen	2005	China	Chin J Arterioscler	PCR-RFLP	rs3918242 (*P*_HWE_ = 0.17)	78 (male = 57, female = 21)	81 (male = 58, female = 23)	Blood
Meng	2006	China	Tianjin Med J	PCR	rs3918242 (*P*_HWE_ = 0.99)	59 (male = 19, female = 40)	99 (male = 32, female = 67)	Blood
Nuzzo	2006	Sicily	Ann N Y Acad Sci	PCR	rs3918242 (*P*_HWE_ = 0.18)	115 (male = 109, female = 6)	123 (male = 100, female = 23)	Blood
Wang	2007	China	Journal of Clinical Hematology	PCR-RFLP	rs3918242 (*P*_HWE_ = 0.27)	37 (male = 29, female = 8)	84 (male = 52, female = 32)	Blood
Horne	2007	America	Am Heart J.	TaqMan	rs3918242 (*P*_HWE_ = 0.34)	1693	3455	Blood
Koh	2008	South Korea	International Journal of Cardiology	PCR-RFLP	rs3918242 (*P*_HWE_ = 0.20)	206	173	Blood
Ma	2010	China	Chin J Hypertens	PCR-SphI	rs3918242 (*P*_HWE_ = 0.70)	362 (male = 249, female = 113)	419 (male = 292, female = 127)	Blood
J.M.	2016	Mexico	Genetics and Molecular Research	PCR-RFLP	rs3918242 (*P*_HWE_ = 0.67)	236 (male = 194, female = 42)	285 (male = 134, female = 151)	Blood
EI-Aziz	2017	Egypt	International Journal of Cardiology	PCR-RFLP	rs3918242 (*P*_HWE_ = 0.69)	184 (male = 150, female = 34)	180 (male = 155, female = 25)	Whole blood
Abdolreza Daraei	2017	Iran	Genetic Testing and Molecular Biomarkers	PCR-RFLP	rs3918242 (*P*_HWE_ = 0.53)	117 (male = 72, female = 45)	120 (male = 68, female = 52)	Whole blood

SNP = single nucleotide polymorphism; HWE = Hardy-Weinberg equilibrium; *P*_HWE_ = *P* value of Hardy-Weinberg equilibrium test in controls for each locus; PCR = polymerase chain reaction.

## Data Availability

The datasets used and analyzed during the current study are available from the corresponding author on reasonable request.
